# Brusatol Inhibits Proliferation and Metastasis of Colorectal Cancer by Targeting and Reversing the RhoA/ROCK1 Pathway

**DOI:** 10.1155/2022/7132159

**Published:** 2022-05-18

**Authors:** Rui-jin Lu, Guo-zhi Zhao, Rong Jiang, Shuang He, Hang Xu, Jia-ming He, Yue Sun, Meng-na Wu, Jian-hua Ran, Di-long Chen, Jing Li

**Affiliations:** ^1^Lab of Stem Cell and Tissue Engineering, Department of Histology and Embryology, Chongqing Medical University, Chongqing, China; ^2^Department of Urology, The First Affiliated Hospital of Chongqing Medical University, Chongqing, China; ^3^Neuroscience Research Center, College of Basic Medicine, Chongqing Medical University, Chongqing, China; ^4^Chongqing Key Laboratory of Development and Utilization of Genuine Medicinal Materials in Three Gorges Reservoir Area, Chongqing, China

## Abstract

Brusatol (BRU) is an important compound extracted from Brucea javanica oil, whose pharmacological effects are able to induce a series of biological effects, including inhibition of tumor cell growth, anti-inflammatory, antiviral, and antitumor. Currently, there are so few studies about the brusatol effects on colorectal cancer that its anticancer mechanism has not been clearly defined. In this study, we made an in-depth investigation into the brusatol effect towards the proliferation and metastasis of colon cancer and the possible mechanism. The inhibitory effect of BRU on the proliferation of colorectal cancer cells was unveiled via CCK-8 method and colony formation assay, while the inhibitory effect of BRU on migration and invasion of colorectal cancer cells was revealed by scratch assay and transwell assay. In addition, Western blot results also revealed that BRU inhibited not only the expressions of RhoA and ROCK1 but also the protein expressions of EMT-related markers e-cadherin, N-cadherin, Vimentin, MMP2, and MMP9 in colon cancer cells. Through the xenotransplantation model, our in vivo experiment further verified the antitumor effect of BRU on colon cancer cells in vitro, and the results were consistent with the protein expression trend. In conclusion, BRU may inhibit the proliferation and metastasis of colorectal cancer by influencing EMT through RhoA/ROCK1 pathway.

## 1. Introduction

Colorectal cancer (CRC) is one of the most common gastrointestinal malignancies, causing nearly 700,000 deaths every year, and is the fourth fatal cancer in the world. The incidence of colorectal cancer has increased over the past decade, and while the use of many emerging chemotherapy drugs has increased the average survival time for patients with advanced colorectal cancer, patients usually die within three years [1]. The five-year survival rate for patients with advanced colon cancer is reported to be less than 10%[2], and there are about 20% and 30% of CRC patients diagnosed with remote metastases on their first visit [3, 4]. Metastasis is the primary cause of death in solid tumors [5], as is colorectal cancer. At present, the treatment of colorectal cancer is mainly surgery-based comprehensive treatment, but postoperative recurrence and metastasis are still the main cause of death of colorectal cancer patients. In the treatment of metastatic colorectal cancer, cetuximab and other drugs have achieved good clinical efficacy but are prone to drug resistance [6, 7]. Poor treatment outcomes highlight the need for a better understanding of the mechanisms that contribute to the onset, development, metastasis, and spread of colorectal cancer.

Metastasis is a multifactorial and multicellular process involving the dynamic formation and breakdown of actin structures [8]. Rho GTplase is one of the most important protein families regulating cell migration, playing a crucial role in regulating cell morphology, motility, cell-cell, and cell-matrix adhesion [9].

Rho kinase (ROCK) is a key serine/threonine kinase downstream of Rho, and the activated RhoA activates ROCK1, leading to the inactivation of myosin phosphatase due to phosphorylation and then resulting in the failure of dephosphorylation of phosphorylated myosin, which would ultimately increase the content of the phosphorylated myosin in cytoplasm and incur more interaction between actin and myosin, thereby the cell adhesion, invasion, and migration are brought about ^[^10, 11]. ROCK is deemed as an anticancer target for its role in promoting the invasion and migration of various cancers [12–14].

Brusatol (BRU) is a bioactive triterpenoid extracted from Brucea javanica oil. It also has a variety of biological effects, including inhibiting tumor cell growth, reducing malaria site replication, reducing inflammation, and resisting virus invasion [15, 16].

At present, BRU has been recognized as an effective antitumor agent for a wide range of tumor cells [15]. Previous studies have shown that BRU would inhibit c-myC synthesis and effectively cripple down tumor cell metabolism and lymphocytic leukemia cell proliferation [17]. Subsequent studies have found that BRU causes rapid and even instantaneous depletion of Nrf2 protein through the posttranscriptional mechanism, thus playing a significant inhibitory effect on the proliferation of HCC cells [18]. At present, it has been pointed out that brusatol, the traditional Chinese medicine, has inhibitory effects on a variety of tumors like liver cancer [19], pancreatic cancer [20], nasopharyngeal carcinoma [21], and melanoma [22]. However, there are few reports about brusatol on colorectal cancer, and its mechanism of action has not been clearly described. Therefore, we made an investigation in this paper into the effects of brusatol on proliferation, migration, and invasion of colorectal cancer cells and then elucidated its role in RhoA/ROCK1 pathway.

## 2. Materials and Methods

### 2.1. Reagents and Antibodies

BRU (14907-98-3, purity > 98%) was fetched from Shanghai Yuanye Biotechnology Co., Ltd. (Shanghai, China), which was dissolved with dimethyl sulfoxide (DMSO) and stored at -80°C. In our subsequent experiments, the BRU was diluted with fresh Dulbecco's Modified Eagle's medium (DMEM, C11995500BT, Gibco) until the final concentration of DMSO was less than 0.1%. MMP2 (40994S), MMP9 (13667S), and E-cadherin (14472S) were purchased from Cell Signaling Technology, USA. Vimentin (AF0318), N-cadherin (AF0243), RhoA (AF2179), ROCK1 (AF1795), and the ROCK inhibitor (Y37632) were brought from Shanghai Biyuntian Biotechnology Co., Ltd.

### 2.2. Cell Culture and Culture Condition

Human colon cancer cell lines HCT-116 and SW480 were provided by Zhongqiao Xinzhou Biotechnology Company (Shanghai, China). NCM460 human normal colonic epithelial cells were stored in the human tissue embryonic stem cell laboratory of Chongqing Medical University. Those cells were cultured with the 10%-fetal-bovine-serum DMEM medium supplemented (10270-106, Gibco) with 1% penicillin and streptomycin (Beyotime, China) and grown at 5% CO_2_ and 37°C.

### 2.3. Cell Viability Assay

In this experiment, Cell Counting Kit-8 (CCK-8, MedChemExpress, USA, HY-K0301) was used to estimate cell viability. NCM460, HCT-116, and SW480 cells at logarithmic phase were taken, and the cell number was adjusted to 5 × 10^3^/well; the cells were laid in a 96-well cell culture plate; then, 100 *μ*L of medium was added to each well. After the cellular adherence, the cells were treated with 0-160 nM BRU for 24, 48, and 72 h, respectively. Then, we added 10 *μ*L of CCK-8 to each well and incubated the cells for 2 hours. The absorbance of each well was measured at 450 nm by a microplate reader (Bio-Rad, CA, USA). Finally, we used the GraphPad Prism 8 software to reckon the BRU's effects at different concentrations on the IC50 of HCT-116 and SW480 cells. The experiment was repeated three times.

### 2.4. Cell Colony Formation Assay

HCT-116 and SW480 cells of logarithmic growth stage were inoculated into 6-well plates with 2 × 10^2^ cells per well. After the cellular adherence, the cells were treated with or without BRU for 24 h. After that, the culture medium was replaced with fresh DMEM, and the cells were continued to be cultured for another two weeks. The cells were then fixed with 4% paraformaldehyde for 20 min at room temperature, then washed with PBS, and stained with 1% crystal violet solution (Beyotime, China). Finally, the ImageJ software was used to take photos and reckon the data. The experiment was repeated three times.

### 2.5. Wound-Healing Assay

HCT-116 and SW480 cells were inoculated into 6-well plates at a density of 5 × 10^4^/mL. After the cells were fully grown, a straight line was scratched in the central area of cell monolayers with sterilized 200 *μ*L head. Subsequently, the cells were washed by PBS and incubated in serum-free DEME with or without BRU. Then, a random plate of cells was taken from each group and observed and photographed under an inverted microscope immediately after the scratches. The remaining cells were incubated in a 5% CO_2_ incubator at 37°C for 24 h and observed under an inverted microscope. Five fields were randomly selected to be taken photos of. The ImageJ software was used to calculate the areas of the scar and the relative mobility of each group. The experiment was repeated three times.

### 2.6. Transwell Assay

Matrigel (Corning, USA, 356234) gel was diluted with serum-free DEME medium in the ratio of 8 ∶ 1 and thoroughly mixed. The mixture was evenly spread over a Transwell upper chamber with pore diameter of 8.0 *μ*m (Corning, USA, 3422), 100 *μ*L per well. The plates were placed at 37°C for 4 h until the gel was solidified. Each well of the Transwell upper chamber was inoculated with 5 × 10^4^ HCT-116 and SW480 cells with the serum-free DMEM medium containing different final concentrations of BRU added into. 500 *μ*L DMEM medium (containing 20% fetal bovine serum) was added to the lower chamber of each well; then, the plates were incubated in incubators for 24 h. After that, noninvasive cells in the upper chamber were gently wiped with cotton. The bottom of the chamber was fixed with 4% paraformaldehyde at room temperature for 15 min. After washing with PBS, the cells stained with 1% crystal violet solution, and 5 fields of view were randomly selected from each group under the microscope to observe and taken pictures of. The experiment was repeated three times.

### 2.7. Western Blot Assay

Tumor samples from tumor cells or homogenates were cleaned with PBS and suspended again in a lysate containing 1% phenyl-methane-sulfonyl fluoride (Beyotime, China) before use. After standing on ice for 30 min, the supernatant was collected after centrifugation at 12 000 rpm at 4°C for 15 min, and the protein concentration was determined using BCA protein detection kit (Beyotime, China). After SDS-PAGE treatment, the isolated proteins were transferred onto polyvinylidene fluoride (PVDF) membrane. The membranes were blocked with rapid blocking solution (New Cell&Molecu biotech, China) at room temperature for 15 min, incubated with corresponding primary antibody overnight at 4°C, washed in Tris-buffered saline with Tween 20 (TBST) for 30 min, and incubated with corresponding secondary antibody for 1 h at room temperature. Bound immune-complexes were detected by hypersensitive enhanced chemiluminescence (ECL) solution (Biosharp, China) and visualized them by luminescence image analyzer (Bio-Rad, CA, USA). The experiment was repeated three times.

### 2.8. Immunofluorescence Staining

The cells were treated with BRU for 24 h and then fixed with 4% paraformaldehyde at room temperature, permeabilization with 0.5% Triton X-100 in PBS for 20 min and then incubated with 1% goat serum albumin blocking solution. Finally, corresponding primary antibodies were added in the cells and incubated overnight at 4°C. After being washed thrice with PBS, the cells were incubated with FITC-conjugated secondary antibodies at 37°C for 1 h. At the last 5 min, the nuclei were stained with DAPI. Images were captured by fluorescence microscope (Olympus, Japan). The experiment was repeated three times.

### 2.9. Q-PCR (Quantitative Real-Time PCR) Assay

HCT-116 cells were collected after treated with or without 6 nM BRU for 24 h. Total RNA was extracted with TRIzol reagent (Invitrogen, Carlsbad, CA). RNAs were converted to cDNAs using a reverse transcription kit (Takara, Japan), SYBR® Select Master Mix (2X) (ABI, USA) to measure mRNA expressions, and the mRNAs were quantified through -*ΔΔ*Ct method. Primer sequences used in this experiment were as follows:

RhoA (forward): GGAAAGCAGGTAGAGTTGGCT

RhoA (reverse): GGCTGTCGATGGAAAAACACAT

ROCK1 (forward): AAGTGAGGTTAGGGCGAAATG

ROCK1 (reverse): AAGGTAGTTGATTGCCAACGAA

### 2.10. Xenograft Models in Nude Mice

BALB/C nude mice (female, 5 weeks old) were purchased from Beijing Vital River Laboratory Animal Technology Co., Ltd. After being fed for 1 week in animal Experiment Center of Chongqing Medical University, the nude mice were randomly divided into two groups. And 0.2 mL HCT-116 cell suspension (1 × 10^7^ cells/mL) was subcutaneously injected into the right axilla of nude mice. When the tumors grew to 0.5 cm in diameter, the mice were randomly divided into two groups. Mice in the treatment group were intraperitoneally injected with 2 mg/kg BRU, and mice in the control group were intraperitoneally injected with normal saline once every two days for 28 consecutive days. Parameters of animal weights and tumor sizes were recorded before each administration. After treatment, the animals were sacrificed; all tumors were isolated and weighed. The tumor volume was calculated through the formula (length × width^2^/2). Nude mice were injected with 0.2 mL HCT-116 cell suspension (1 × 10^7^ cells/mL) through tail vein and randomly divided into two groups: BRU group was injected intraperitoneally with 2 mg/kg BRU once every two days, and the control group was injected intraperitoneally with normal saline. After 28 days of treatment, the mice were sacrificed, and the metastatic nodules in lung and intestine were counted. All animal experiments were approved by the Animal Experiment Center of Chongqing Medical University and carried out in accordance with the principles of animal care.

### 2.11. HE Staining

Xenograft tumor tissues from different groups were fixed with 10% neutral buffer formalin, embedded in paraffin, and sectioned with the thickness of 8 *μ*m. The sections were then stained with a HE assay kit (Solarbio, China) according to the manufacturer instructions. Histological observation was conducted with light microscope (×200 and ×400; Nikon).

### 2.12. Statistical Analysis

Data in this paper were displayed in a manner of mean ± SD (standard deviation). Statistical analysis was performed with the GraphPad Prism 8.0 software (San Diego, CA, USA), and the data significance was analyzed via either *t*-test or bidirectional analysis of variance (ANOVA).

## 3. Results

### 3.1. BRU Inhibited Both the Proliferation of HCT-116 and SW480 Cells

The chemical structure formula of BRU (C_26_H_32_O_11_) was shown in Figure 1(a). HCT-116 cells and SW480 cells were treated with different concentrations of BRU for 24, 48, and 72 h, and the cell viability was detected by CCK-8 method, so that we could determine the effects of BRU on the proliferation of colorectal cancer cells in vitro. And it turned out that BRU significantly inhibited the proliferation of HCT-116 cells and SW480 cells in a dose-dependent and time-dependent manner (Figures 1(c) and 1(d)). Normal colonic epithelial cell line NCM460 was treated with BRU at the same low concentration, and no toxicity of BRU to NCM460 cells was detected by cell viability tests (Figure 1(b)). The IC_50_ of HCT-116 and SW480 cells was 16.63 nM and 76.07 nM, respectively, after treated with BRU for 24 h, while the survival rate of the two cells was more than 90% when treated with 20 nM and 80 nM BRU for 24 h. Therefore, unless otherwise specified, we continued to treat HCT-116 and SW480 cells with 20 nM and 80 nM BRU as the maximum concentration, and 24 h was the treatment duration.

In the colony formation experiment, we selected the concentration of IC_50_ and 1/2 IC_50_ about 24 h after BRU acted on HCT-116 and SW480 cells to treat the cells, so as to explore the effect of BRU on the proliferation of CRC cells. The results showed that BRU significantly reduced the colony-forming ability of colorectal cancer cells, and the inhibition effect was most significant in the highest concentration group (Figures 1(e)–1(h)). These results all confirmed the inhibitory effect of BRU on the proliferation of CRC cells in vitro.

### 3.2. BRU Inhibited Both the Migration and Invasion of HCT-116 and SW480 Cells In Vitro

This section investigated the effects of BRU on migration and invasion of HCT-116 and SW480 cells. We treated HCT-116 and SW480 cells with increasing concentrations of BRU for 24 h and found that BRU significantly inhibited the migration and invasion of HCT-116 (Figures 2(a) and 2(e)) and SW480 (Figures 2(c) and 2(g)) cells. In HCT-116 cells, the relative mobility of each group was (28.9 ± 0.8)%, (17.7 ± 1.6)%, and (10.3 ± 3.1)% (Figure 2(b)); through calculation, we learned that the number of invaded membrane cells in each group was 760 ± 27, 532 ± 57, and 353 ± 8 under each field (Figure 2(f)). In SW480 cells, the relative mobility of each group were (59.1 ± 3.8)%, (22.8 ± 2.3)%, and (7.4 ± 3.1)% (Figure 2(d)); after calculation, the number of invaded membrane cells per field of vision in each group was 926 ± 99, 676 ± 19, and 608 ± 8 (Figure 2(h)).

### 3.3. BRU Reversed the Epithelial-Mesenchymal Transformation (EMT) of HCT-116 and SW480 Cells

EMT is involved in the migration and invasion of most malignant tumor cells [23]. We treated HCT-116 and SW480 cells with BRU (0, 3, and 6 nM) and BRU (0, 10, and 20 nM) for 24 h, respectively, and detected EMT-related proteins expression by western blot. The results showed that compared with the control group, the expression of E-cadherin protein was upregulated in both HCT-116 and SW480 cells treated with BRU, while the expressions of Vimentin, N-cadherin, MMP2, and MMP9 protein were downregulated (Figures 3(a)–3(d)).

### 3.4. BRU Inhibited Colorectal Cancer Cellular Invasion by Blocking the RhoA/ROCK1 Pathway

HCT-116 and SW480 cells were treated with BRU (0, 3, and 6 nM) and BRU (0, 10, and 20 nM), respectively, to verify the antitumor mechanism of BRU on colorectal cancer cells. After 24 h treatment, the expressions of RhoA/ROCK1 pathway protein were assessed by western blot assay. Western blot results showed that compared with the control group, protein expressions of RhoA and ROCK1 in both HCT-116 (Figures 4(a) and 4(c)) and SW480 (Figures 4(b) and 4(d)) cells were significantly reduced in a concentration-dependent manner after BRU treatment. In addition, the immunofluorescence results of HCT-116 cells after 6 nM BRU treatment showed that the protein expressions of RhoA and ROCK1 in the BRU treatment group were greatly decreased in contrast to the control group (Figures 4(e) and 4(f)). Likewise, q-PCR results unveiled that the mRNA expressions of RhoA and ROCK1 were also decreased after BRU treatment (Figure 4(g)).

### 3.5. BRU Reversed the EMT Process of HCT-116 and SW480 Cells by Blocking RhoA/ROCK1 Signaling Pathway

Subsequent experiments verified that BRU affects the EMT process of colorectal cancer cells through RhoA/ROCK1 signaling pathway: we treated HCT116 and SW480 cells with BRU, Y27632 (inhibitors of ROCK), and BRU + Y27632. The protein expression levels of RhoA, ROCK1, E-cadherin, Vimentin, N-cadherin, MMP2, and MMP9 were detected by western blot. The results showed that BRU inhibited the expressions of RhoA and ROCK1 proteins in both HCT-116 and SW480 cells. In addition, Y27632 also downregulated the levels of these proteins, and BRU enhanced the downregulation of these proteins by Y27632 (Figures 5(a)–5(d)). In Figures 5(e)–5(h), HCT-116 and SW480 were treated in the same way, and the results showed that both BRU and Y27632 could enhance the protein expression of E-cadherin and inhibit the protein expressions of Vimentin, N-cadherin, MMP2, and MMP9. Moreover, the BRU + Y27632 treatment group enhanced or inhibited the expression of these proteins more significantly. Together, these results implied that BRU reverses EMT in colorectal cancer cells by blocking the RhoA/ROCK1 pathway.

### 3.6. BRU Inhibited Tumor Growth and Metastasis in HCT-116 Xenograft Mice

The mouse HCT-116 xenotransplantation model was used to study the antitumor effect of BRU in vivo. In order to investigate whether BRU inhibits tumor growth in vivo, the HCT-116 cells were inoculated subcutaneously into nude mice to construct mouse models. These mice were divided into control group and BRU group. It was seen that the tumor volume in the BRU group was significantly smaller than that in the control group (Figure 6(a)), and its weight was also significantly lighter (Figure 6(e)). In addition, our outcomes of measurements showed that at the beginning of administration, the tumor volume of the control group and the BRU group was almost the same. With the increase of administration time, the tumor volume of the control group increased, while that of the BRU group did not change much (Figure 6(d)). There was no significant difference in mouse body weight between control and BRU groups, suggesting that BRU has no toxic side effects (Figure 6(b)).

In addition, paraffin-embedded sections of tumor tissues were analyzed by HE staining, and it was observed under ×200 and ×400 microscopes that tumor tissue necrosis, nuclear fragmentation, and dissolution were evident in the BRU group versus the control group (Figure 6(c)). Western blot analysis of tumor tissue showed that the expressions of RhoA, ROCK1, Vimentin, N-cadherin, MMP2, and MMP9 protein decreased, and the expressions of E-cadherin protein increased (Figures 6(f) and 6(g)), which was consistent with the results of in vitro experiment.

In the early stage of treatment, the weight of mice in each group was not significantly different; but in the late stage of treatment, that is, three weeks after the drug was administered, due to the massive proliferation and metastasis of tumor cells, the body weight of the mice in the control group decreased significantly. The body weight of the mice in the two groups was almost unchanged, and the body weight of the two groups of mice was significantly different, and the difference was statistically significant (Figure 6(h)). We then counted metastatic nodules in the lung and intestine, and the results showed that the number of metastatic nodules in the lung and intestine was significantly reduced by more than 60.8% and 57.1% compared with the control group (Figures 6(i) and 6(j)). These results suggest that BRU is capable of inhibiting the growth and metastasis of colorectal cancer cells in vivo.

## 4. Discussion

One of the merits of Chinese herbal medicine is less toxic and side effects, which has been coming to be concerned last decades, especially in antitumor realm. Brusatol, one of the herbal extracts, has been widely recognized for its remarkable efficacy in the treatment of many cancer diseases [24, 25]. Our studies found that BRU has a significant inhibitory effect on the growth of colorectal cancer cells in both vivo and vitro, which also indicates that BRU has potential clinical application value in the development of new remedies for CRC.

The proliferation ability of tumor cells is the basis of tumor growth and development, and all tumors have the distinctive characteristic of uncontrolled proliferation [26]. Our study verified the effective inhibitory effect of BRU on the proliferation of HCT-116 cells and SW480 cells. We conducted CCK-8 analysis and colony formation test successively and found that BRU reduced the growth capacity of HCT-116 cells and SW480 cells in a time-dependent and dose-dependent manner. In addition, the number of cell colonies formed in treatment group was significantly less than that in the control group. The results above all reflected the inhibitory effect of BRU on CRC cellular proliferation in vitro.

The process of tumorous metastasis is not only complex but also a malignant behavior in the occurrence and development of tumor. Migration and invasion are two essential cellular processions in tumor metastasis [27]. Both scratch assay and Transwell assay results showed that BRU effectively inhibited the migration and invasion of HCT-116 and SW480 cells in a dose-dependent manner, which was sufficient to demonstrate the effective inhibitory effect of BRU on the migration and invasion of CRC cells.

EMT is a morphogenetic process, which also occurs in cancer, triggering loss of cell polarity, disruption of cell-cell adhesion, actin cytoskeletal recombination, and cell migration. The transformation of cells with an epithelial phenotype into cells with a mesenchymal phenotype is called epithelial-mesenchymal transformation, a normal process required for embryonic development and one of the pathologic features associated with tumor metastasis [28]. EMT plays a crucial role in early tumor metastasis, enabling tumor cells to migrate and invade and at the same time giving tumor cells the properties of stem cells [29, 30]. Among the markers of EMT, high expression of N-cadherin is positively correlated with HCC and colon cancer tissue metastasis, suggesting a low survival rate in patients [31]. Vimentin is commonly expressed in nondiseased mesenchymal cells and overexpressed in a wide range of epithelial cancers, which are also positively associated with tumor proliferation, metastasis, and reduced patient survival [32]. Reduction of E-cadherin is associated with invasion of CRC cells, and it would also increase the tumor cellular resistance to standard chemotherapy drugs [33, 34]. MMP2 enhances fibronectin mediated tumor cell adhesion by regulating the migration of various tumor cells in the extracellular matrix through integrin [35]. MMP9 is able to effectively affect the vascularization and growth rate of tumor cells, leading to the formation and degradation of cell-matrix [36]. Therefore, reversing the procession of EMT is considered as a potential strategy to improve the migration and aggressiveness of malignant tumors. Western blot assay revealed that BRU inhibits the EMT of cancer cells by upregulating the expression of E-cadherin and downregulating the protein levels of Vimentin, N-cadherin, MMP2, and MMP9, thus hindering the metastasis of colon cancer cells.

Cancer cell migration is a multistep dynamic process involving cell-cell adhesion, cell-matrix adhesion, and biochemical and biophysical reorganization of cell shape or polarity [37, 38], and one of the key requirements of tumor metastasis is the recombination of actin cytoskeleton. Actin is the critical component of cytoskeleton, the main mediator of intercellular force generation, and it is also the key component of cell diffusion and adhesion. Cytoskeletal recombination of actin is also essential for the transition of adequately characterized epithelial-mesenchymal transition (EMT) to mesenchymal like cells [39]. Studies have shown that RhoA-ROCK1 signaling pathway is related to cytoskeleton regulation, which has an important impact on cancer metastasis [40]. Studies have also justified that targeting RhoA-ROCK1 signaling pathway is one of the feasible methods to inhibit CRC metastasis [41]. A study on colon cancer cells showed that expression and subsequent activation of RhoC protein, accompanied with the downregulation of E-cadherin and a significant reduction in RhoA activation, are associated with EMT development [42]. Therefore, we have reason to believe that BRU would inhibit EMT through RhoA/ROCK1 pathway, thus inhibiting the proliferation and metastasis of colorectal cancer. In this study, we found that the protein and mRNA expressions of RhoA and ROCK1 were decreased in BRU-treated colorectal cancer cells. After the addition of ROCK1 inhibitor (Y27632) to inhibit ROCK1 expression, BRU would further enhance the inhibitory effect of Y27632 on colorectal cancer cells.

In addition, our in vivo experiments further confirmed the antitumor effect of BRU. These findings suggested the antiproliferation and antimetastasis effects of BRU towards CRC, which may be related to the reversal of EMT by targeting the RhoA/ROCK1 pathway.

## 5. Conclusion

In summary, this study for the first time clarified the anticolorectal cancer role of BRU: BRU inhibits tumor growth and metastasis in vivo and in vitro by blocking the RhoA/ROCK1 signaling pathway-mediated EMT process. These findings provide solid evidence that BRU may be an attractive candidate for the treatment of CRC in the future. However, tumor metastasis is a complex process, and whether BRU regulates this process through other mechanisms is worthy of our further exploration.

## Figures and Tables

**Figure 1:** BRU inhibited the proliferation of HCT-116 and SW480 cells in vitro. Chemical structures of BRU (a), NCM 460 (b), HCT-116 (c), and SW480 (d) cells were treated with various specified concentrations of BRU (0-160 nM) for 24, 48, and 72 h, respectively, and cell viability was measured by CCK-8 assay. Images were formed of representative colonies of HCT-116 cells (e) and SW480 cells (f) treated with different concentrations of BRU. (g, h) Statistical analysis of cell colony formation of HCT-116 and SW480. All data were shown as mean ± SD from three independent trials (^∗^*P* < 0.05, ^∗∗^*P* < 0.01 vs. control).

**Figure 2:** BRU inhibited the migration and invasion of HCT-116 and SW480 cells. Wound healing experiments were performed to detect representative images (a, c) and statistical analysis of cell mobility (b, d) of HCT-116 and SW480 cells treated with different concentrations of BRU for 24 h. Representative images (e, g) of the invasion results of HCT-116 and SW480 cells treated with BRU at different concentrations were detected by transwell assay. Statistical plots of invaded cells (f, h). All data were shown as mean ± SD from three independent trials (^∗^*P* < 0.05, ^∗∗^*P* < 0.01 vs. control).

**Figure 3:** BRU reversed protein expressions of EMT-related markers in both HCT-116 and SW480 cells. Western blotting was performed to analyze the protein level of E-cadherin, Vimentin, N-cadherin, MMP9, and MMP2 in HCT-116 cells (a, b) and SW480 cells (c, d), and quantitative analysis was performed by the Image Lab software. All data were shown as mean ± SD from three independent trials (^∗^*P* < 0.05, ^∗∗^*P* < 0.01 vs. control).

**Figure 4:** BRU downregulates RhoA/ROCK1 pathway protein expressions in colorectal cancer cells. After the respective treatment concentrations were added into HCT-116 and SW480 cells, the expressions of RhoA and ROCK1 in the treated and the untreated groups were detected by western blot (a, b), and the results of quantitative analysis by the Image Lab software (c, d). Representative immunofluorescence images of HCT-116 cells treated with or without 6 nM BRU for 24 h (e, f). The mRNA expressions of RhoA and ROCK1 in HCT-116 cells were determined by RT-QPCR (g). All data were shown as mean ± SD from three independent trials (^∗^*P* < 0.05, ^∗∗^*P* < 0.01 vs. control).

**Figure 5:** Possible mechanism of BRU reversal of EMT process in colorectal cancer cells. After HCT-116 and SW480 cells were treated with or without BRU, Y27632 and BRU + Y27632, RhoA and ROCK1 in cells were analyzed by western blot (a, c) and quantitative analysis by the Image Lab software (b, d); after HCT-116 and SW480 cells were treated with or without BRU, Y27632, BRU + Y27632, western blot analysis of E-cadherin, Vimentin, N-cadherin, MMP2, MMP9 in cells (e, g) and quantitative analysis of the Image Lab software (f, h). All data were shown as mean ± SD from three independent trials (^∗^*P* < 0.05, ^∗∗^*P* < 0.01 vs. control).

**Figure 6:** BRU inhibits the tumorous growth and metastasis in nude mice. Representative image of nude mouse tumor in subcutaneous tumor-forming model of the control group (normal saline) and BRU (2 mg/kg) group (a). Changes in body weight of mice in the control group and BRU group during treatment (b). Representative image of HE staining in tumor tissue (c). Changes in tumor volume and weight were compared between the control group and the BRU group during treatment (d, f). The protein levels of RhoA, ROCK1, E-cadherin, Vimentin, N-cadherin, MMP2, and MMP9 in tumor tissues were analyzed by western blotting (g, h). Body weight changes of the control group and BRU group in the nude mouse model after tail vein injection (h). Metastatic nodules in lung and bowel (i, j). All data were shown as mean ± SD from three independent trials (^∗^*P* < 0.05, ^∗∗^*P* < 0.01 vs. control).

## Data Availability

The data used to support the findings of this study are included within the article.
